RETRACTED

# Analysis on Effects of Laparoscopic Total Hysterectomy Combined with High Hysterosacral Ligament Suspension in the Treatment for Uterine Prolapse

**DOI:** 10.1155/2022/2585529

**Published:** 2022-08-29

**Authors:** Bing Qiu, Aili Wang, Yanxin Chen, Zhijun Wang

**Affiliations:** ^1^Haikou Hospital of Traditional Chinese Medicine, No. 45, Jinpan Road, Haikou 570216, Hainan, China; ^2^The 928th Hospital of the Joint Logistics Support Force of the Chinese People's Liberation Army, No. 100, Longkun South Road, Haikou 570216, Hainan, China

## Abstract

**Objective:**

To investigate the effect of laparoscopic total hysterectomy combined with high hysterosacral ligament suspension on the treatment for uterine prolapse.

**Methods:**

A total of 100 patients with uterine prolapse treated in our two hospitals from January 2019 to December 2021 were included in this study, which were divided into two groups through the number double-blind method, with 50 patients in each group. The control group was treated with transvaginal total hysterectomy, and the research group was treated with laparoscopic total hysterectomy combined with high hysterosacral ligament suspension. The surgical effect on patients was evaluated through the pelvic organ prolapse quantification method (POP-Q). The patients' adverse reactions were compared. The quality of sexual life was evaluated with the short form of the pelvic organ prolapse/urinary incontinence sexual questionnaire (PISQ-31). And, the patients' quality of life was also evaluated with the pelvic floor distress inventory-short form 20 (PFDl-20).

**Results:**

The surgical effect on the control group and the research group was 80.00% and 96.00%, respectively, with statistical significance (*X*^2^ = 6.601, *P* < 0.001). The incidences of adverse reactions of the two groups were 4.00% and 6.00%, respectively, which were comparable (*X*^2^ = 0.211, *P* =  0.646). The total PISQ-31 scores before surgery of the control group (97.07 ± 9.80) and the research group (97.02 ± 9.80) were comparable (*t* = 0.020, *P* = 0.984), and those after surgery were 112.55 ± 13.78 in the control group and 130.80 ± 17.42 in the research group, respectively, with statistical significance (*t* = 4.500, *P* < 0.001). And, the total PFDl-20 scores before surgery of the control group (72.50 ± 13.58) and the research group (72.50 ± 13.60) were comparable (*t* = 0.057, *P* = 0.098), and that after surgery were 56.10 ± 10.51 in the control group and 42.30 ± 8.05 in the research group, respectively, with statistical significance (*t* = 5.709, *P* < 0.001).

**Conclusion:**

Laparoscopic total hysterectomy combined with high hysterosacral ligament suspension has an ideal effect in patients with uterine prolapse, with few adverse reactions, effectively promoting the improvement of the quality of patients' sexual life and their life. This combination has the significance of active promotion in the clinic.

RETRACTED

## 1. Introduction

Uterine prolapse is a common disease of pelvic organ prolapse clinically in gynaecology. The disease is manifested by uterine tissues descending around the vaginal axis, the level of the external os of cervix being the same as or lower than the ischial spine, and the cervix and uterine body all prolapsing out of the orificium vaginae [1]. The majority of patients with uterine prolapse are middle-aged and elderly females, with a high incidence. Mild uterine prolapse has no obvious clinical symptoms, but when the disease develops to moderate or severe, it will seriously affect the quality of patients' daily life [2, 3]. Related studies showed that [4] although transvaginal total hysterectomy has an ideal effect in patients with uterine prolapse but no willingness to retain the uterus, the prognosis is poor. With the rapid and continuous development of medical science and technology in China, laparoscopic technology has been widely used in clinical practice. And, laparoscopic high uterosacral ligament suspension is more safe and reliable for uterine prolapse [5, 6]. On account of this, our two hospitals performed laparoscopic total hysterectomy combined with high hysterosacral ligament suspension for patients with uterine prolapse but no willingness to retain the uterus, which had an ideal effect. The research process is reported as follows:

## 2. Data and Methods

### 2.1. General Data

A total of 100 patients with uterine prolapse treated in our two hospitals from January 2019 to December 2021 were included in this study, which were divided into two groups, control group and research group, through the number double-blind method, with 50 patients in each group. Patient data are shown in Table 1, which were comparable (*X*^2^/*t* = 0.267, 0.407, 0.199, *P* = 0.790, 0.685, 0.843). The study was approved by the ethics committee of our hospital.

### 2.2. Inclusion and Exclusion Criteria

#### 2.2.1. Inclusion Criteria

(1) Patients who had clinical symptoms and signs met the diagnosis criteria of uterine prolapse in obstetrics and gynecology and were admitted to our hospital for surgical treatment [7]; (2) patients who met the indications of laparoscopic total hysterectomy and high hysterosacral ligament suspension; (3) Patients who had complete basic information and volunteered to join the study after understanding the study content.

#### 2.2.2. Exclusion Criteria

(1) Patients with gastrointestinal diseases, liver and kidney dysfunction, urinary system diseases, cervical cancer. (2) Patients with contraindications to surgery or anesthesia. (3) Patients suffering from mental illness, mental disorder, and communication disorder.

RETRACTED

### 2.3. Methods

#### 2.3.1. Preparation before the Surgery

After the patients were admitted to the hospital, the medical staff assisted the patients in completing the blood routine examination, urine and stool, ECG, chest X-ray, abdominal cavity, pelvic color ultrasound, and other related preoperative examinations. For those patients who had other systemic diseases, the corresponding examinations were conducted to control BP and glucose. In the evening of D1 before surgery, the nurse was responsible for routine vaginal scrub and enema preparation for patients, and for those with hypertension, oral antihypertensive drugs were given early in the morning of the day for the surgery.

#### 2.3.2. For the Control Group, Transvaginal Total Hysterectomy Was Performed

The patients were first given general anesthesia in the bladder stone position. For those who had vaginal prolapse, the anterior and posterior vaginal repair was given at the same time. (1) The labium anterius was pulled. According to the instructions of the metal catheter, a surgical incision was made 5 mm below the junction of bladder and cervix, for circumcision from mucous membrane to cervical fascia, and a blunt-sharp separation was performed in the space between bladder and cervix fascia. The bladder was pushed up to the reflection of vesicouterine peritoneum. The vesicocervical ligament was clamped with the surgical forceps and cut off. And then, the stumps were sutured. (2) The reflection of vesicouterine peritoneum was lifted and cut, which was marked with sutures. The cervix was pulled forward, and blunt-sharp dissection was made bilaterally at the posterior fornix. After the rectum was pushed away, the uterorectal peritoneum was lifted. After reflexing, the uterorectal peritoneum was opened by cutting with surgical scissors and marked with sutures. After blunt-sharp separation, it was clamped with forceps and cut off, and the stumps were sutured. (3) The bilateral cardinal ligaments were clamped in divided fashion, and the stumps were sutured after transection. (4) Uterine arterioveins were clamped with forceps along bilateral walls of the uterus, and the stumps were sutured after transection. After an anterior uterine wall was clamped, the uterus was everted from the pelvic cavity. Bilateral round ligaments, proximal uterine ends of fallopian tubes and ovarian ligaments were cut and sutured, and then, the appendages were inspected bilaterally for abnormalities and stumps for bleeding. (5) The marked sutures were lifted, and the peritoneum was sutured backwards, closing the pelvic peritoneum. After surgery, antibiotics were routinely used to prevent anti-infection prevention and treatment.

RETRACTED

#### 2.3.3. For the Research Group, Laparoscopic Total Hysterectomy Combined with High Hysterosacral Ligament Suspension Was Performed

The patients were first given general anesthesia in the bladder stone position. For those who had vaginal prolapse, the anterior and posterior vaginal repair was given at the same time. (1) After the general anesthesia was success, medical staff established pneumoperitoneum for the patients by making a 10 mm puncture hole at the umbilicus, a 5 mm puncture hole at the McBurney point, a 10 mm puncture hole at the anti-McBurney point, and a 5 mm puncture hole 5 cm to the left of the umbilicus. After the routine vaginal disinfection, the uterine cup was placed and the uterus was pushed up. (2) Bilateral round ligaments were coagulated, and anterior lobes of bilateral broad ligaments were opened. Bilateral isthmus tuba uterinas, ovarian ligament, and infundibulopelvic ligaments were coagulated. Both sides were treated with the correlation method. (3) After the bladder recursion peritoneum was cut, the bladder was pushed down to the external cervical opening, and bilateral uterine arterioles and veins and utero-sacral ligaments were coagulated as well. (4) The uterus was completely removed through the vagina with the uterine cup mouth as the center. (5) The vaginal stump was sutured. The ureter was gradually pushed outward to the lateral peritoneal space as the direction of the ureter, and the fundus ligament tissues were gradually separated. At the point 4 cm from the utero-sacral ligament to the sacrum, No. 2 nonabsorbable suture was used for suturing through folding to the vaginal stump for fixing bilateral sacral ligaments. After surgery, antibiotics were routinely administered to prevent the infection.

### 2.4. Observation Indexes

(1)  The patients were followed up for the first time 3 months after surgery, and for the second time 6 months after surgery, with the success rate of 100%. The contents for following up included clinical symptoms and pelvic cavity examination. The quantification method of pelvic organ prolapse (POP-Q) score was observed and recorded, and the clinical effects of the patients were evaluated according to the POP-Q method. Excellent cases were presented as degree 0, effective cases were presented as degree I, ineffective cases were presented as degrees II and III. The surgical effect was calculated as (number of excellent cases + number of effective cases)/total number of cases × 100%.
  (2)The adverse reactions of the patients were observed and compared: urinary tract infection, urinary retention, and lumbosacral tenesmus.
(3)  Sexual treatment on patients was evaluated with the short form of pelvic organ prolapse—urinary incontinence sexual questionnaire 31 (PFDI-31) before and after surgery. PISQ-31 consists of 31 items in three dimensions: physical status, emotional status, and sexual partner factor. Liket5 scoring method was adopted, which was evaluated from 1 to 5, with the score from 31 to 155. The higher the score, the more ideal the patient's quality of life.
(4)  The patient's quality of life was investigated before and after surgery with the pelvic floor distress inventory questionnaire-20 (PFDI-20). The PFDl-20 questionnaire consists of three evaluation scales, namely, the Pelvic Organ Prolapse Distress Inventory-6 (POPDI-6), the Colorectal-Anal Distress Inventory-8 (CARDI-8), and the Urogenital Distress Inventory-5 (UDI-5), including 20 items in total. Likert 5 scoring method was adopted, which was evaluated from 1 to 4 for this evaluation, with the score from 20 to 80. The higher the score, the more ideal the patients' quality of life.

RETRACTED

### 2.5. Statistical Analysis

The data analysis was performed with statistical software SPSS20.0. Measurement data were represented with $\bar{x}$ ± *s*, and *t*-test was adopted for intergroup comparison. Enumeration data were represented with rate and were tested with *X*^*2*^. *P* < 0.05 was considered that the difference was statistically significant.

## 3. Results

### 3.1. Comparison of Surgical Effects of Patients

The surgical effect was 80.00% of patients in the control group and was 96.00% of patients in the research group, which is statistically significant (*X*^2^ = 6.601, *P* < 0.001), as shown in Table 2.

### 3.2. Comparison of Adverse Effects of Patients

The incidence of adverse reactions was 4.00% in the control group and 6.00% in the research group, which were comparable (*X*^2^ = 0.211, *P*=0.646), as shown in Table 3.

### 3.3. Comparison of the Patient's Sexual Quality of Life

The total score of the two groups were comparable (*P* > 0.05), and the total score of PISQ-31 in the postoperative research group was higher than that of the control group, which was statistically significant (*P* < 0.001), as shown in Table 4.

### 3.4. Comparison of Patient's Quality of Life

The PFDl-20 scores between the two groups were comparable before surgery (*P* > 0.05), but after surgery, the PFDl-20 score of the research group was lower than that of the control group, which was statistically significant (*t* = 5.709, *P* < 0.001), as shown in Table 5.

RETRACTED

## 4. Discussion

The pathogeny of uterine prolapse is more complex, and some patients may develop this disease for a variety of factors, such as genetic tendency, pelvic floor damage during delivery, and connective tissue dysfunction, resulting in a long-term high level of abdominal pressure [8]. Although uterine prolapse does not endanger the patients' life, it has a serious impact on the patients' physiology, psychology, sex, society, and quality of life [9]. At present, patients with uterine prolapse but no willingness to retain the uterus are often treated with transvaginal total hysterectomy in clinic, which has certain effect, but will affect the pelvic supporting structure, resulting in a high incidence of postoperative vaginal dome prolapse. Laparoscopic vaginal sacral fixation has an exact effect and is considered as the gold standard surgery. However, vaginal mesh needs to be implanted in this type of surgery, with higher requirements on the operations of the surgery, and some complications are more serious. Existing clinical studies have found that vascular injury, ureter injury, sacral nerve root injury, and other conditions will occur after surgery [10]. High hysterosacral ligament suspension can reattach the vaginal dome to the high position in the pelvis, simulate the natural attachment point between uterus and sacrum better, and reconstruct the complex of main ligament and hysterosacral ligament, which has been widely used in the treatment for pelvic defects [11].

This study showed that the surgical effect was 80.00% of patients in the control group and was 96.00% of patients in the research group, which is statistically significant (*P* < 0.001). The incidence of adverse reactions was 4.00% in the control group and 6.00% in the research group, which were comparable (*P*=0.646). The results suggest that patients with uterine prolapse treated with laparoscopic total hysterectomy combined with high hysterosacral ligament suspension had similar postoperative complication rate as those who were treated with transvaginal total hysterectomy; however, the former had more ideal effect. According to the analysis, in addition to bleeding and infection, ureteral injury and pelvic nerve root injury are the common complications of uterine prolapse surgery. Although high uterosacral ligament suspension can be performed through the vagina, this type of surgery cannot be regarded as the anatomical marker for ureter, so the risk of ureteral injury is high. Previous clinical studies have shown that [12] the shortest distance between ureter and ipsilateral uterosacral ligament was 13.77 mm, and the ureter was extremely close to the ipsilateral phalanx ligament at 1 cm from the ischial spine to the sacrum. Other studies showed that [13], laparoscopic high sacral ligament suspension can provide high suspension and suture to the uterosacral ligament with the assistance of laparoscopic vision, which can better protect the ureter and pelvic nerve. Meanwhile, this type of surgery can fix the superior standard of the uterosacral ligament, which is safer and more effective compared with the transvaginal method. The treatment combined with high hysterosacral ligament suspension avoids the occurrence of related complications caused by the use of mesh, such as persistent vaginal pain or bleeding, pelvic pain or groin pain, sexual difficulties, or poor quality of life.

RETRACTED

Safe and successful uterine prolapse surgery is not only the smooth progress of hysterectomy and anatomical repair of prolapse, but also the resolution of postoperative symptoms such as intestinal, urinary, and vaginal herniation. In addition, it is necessary to pay attention to the quality of sexual life and quality of life of patients after surgery. At present, there are few reports on the investigation and research of quality of sexual life and quality of life of patients with uterine prolapse after laparoscopic total hysterectomy combined with high hysterosacral ligament suspension in China, most of which only focus on anatomical results [14]. In view of this, in addition to the surgical effect and adverse reactions, the study also included the quality of sexual life and quality of life. This study showed that the difference of PFDl-20 and PISQ-31 scores were comparable between the two groups before surgery (*P* > 0.05), and after surgery, the total PISQ-31 score of the research group was higher than that of the control group, and the PFDl-20 score of the research group was lower than that of the control group, with statistical significance (*P* < 0.001). The results suggest that laparoscopic total hysterectomy combined with high hysterosacral ligament suspension treatment for patients with uterine prolapse, which repair the vaginal dome and maintain it in the normal physical position, can promote the recovery of pelvic floor and bladder function and ameliorate the symptoms of urinary incontinence, lower abdomen tenesmus, and dyspuria caused by the disease, so as to improve patients' sexual function and the quality of life at the same time [15].

In conclusion, laparoscopic total hysterectomy combined with high hysterosacral ligament suspension has an ideal effect in patients with uterine prolapse, with few adverse reactions, which can effectively promote the improvement of quality of sexual life and quality of life of patients. This combination therapy is of positive promotion significance in clinical practice.

RETRACTED

## Figures and Tables

**Table 1:** Comparison of general data of patients ($\bar{x}$ ± *s*).

Group	Number of cases	Age (years old)	Average age (years old)	BMI (kg/m^2^)	Mean BMI (kg/m^2^)	Gravida	Average gravida
Control group	50	40–59	48.10 ± 1.40	20–27	24.80 ± 0.90	1–4	4.10 ± 1.90
Research group	50	40–60	48.00 ± 1.50	20–28	24.70 ± 1.00	1–5	4.00 ± 2.00
*X * ^2^/*t*	—	0.267	0.407	0.199			
*P*	—	0.790	0.685	0.843			

**Table 2:** Comparison of surgical effects of patients (*n*, %).

Group	Number of cases	Number of excellent cases	Number of effective cases	Number of ineffective cases	Number of cases with surgical effect
Control group	50	30 (60.00%)	10 (20.00%)	10 (20.00%)	40 (80.00%)
Research group	50	45 (90.00%)	3 (6.00%)	2 (4.00%)	48 (96.00%)
*X * ^2^	—				6.061
*P*	—				<0.001

**Table 3:** Comparison of adverse reactions of patients (score, $\bar{x}$ ± *s*).

Group	Number of cases	Cases with urinary tract infection	Cases with urinary retention	Cases with lumbosacral tenesmus	Rate of adverse reactions
Control group	50	1 (2.00%)	1 (2.00%)	1 (2.00%)	3 (6.00%)
Research group	50	1 (2.00%)	1 (2.00%)	0 (0.00%)	2 (4.00%)
X^2^	—				0.211
*P*	—				0.646

**Table 4:** Comparison of patients' quality of sexual life (score, $\bar{x}$ ± *s*).

Group	Number of cases	Physical status		Emotional status		Sexual partner factor		Total PISQ-31 score	
		Before surgery	After surgery	Before surgery	After surgery	Before surgery	After surgery	Before surgery	After surgery
Control group	50	48.05 ± 3.20	55.60 ± 5.10	35.72 ± 4.26	39.70 ± 5.23	13.30 ± 2.34	17.25 ± 3.45	97.07 ± 9.80	112.55 ± 13.78
Research group	50	48.01 ± 3.22	64.20 ± 7.10	35.74 ± 4.23	44.45 ± 6.15	13.27 ± 2.35	22.15 ± 4.17	97.02 ± 9.80	130.80 ± 17.42
*t*	—	0.048	5.388	0.018	3.223	0.050	4.959	0.020	4.500
*P*	—	0.962	<0.001	0.986	<0.001	0.961	<0.001	0.984	<0.001

**Table 5:** Comparison of patient's quality of life (score, $\bar{x}$ ± *s*).

Group	Number of cases	POPDI-6 score		Total PFDI-20 score		UDI-6 Score		Total PFDI-20 score	
		Before surgery	After surgery	Before surgery	After surgery	Before surgery	After surgery	Before surgery	After surgery
Control group	50	23.85 ± 4.40	17.50 ± 3.75	26.10 ± 4.28	20.30 ± 2.85	22.55 ± 4.90	18.30 ± 3.91	72.50 ± 13.58	56.10 ± 10.51
Research group	50	23.88 ± 4.38	13.70 ± 2.80	26.11 ± 4.30	15.25 ± 2.50	22.51 ± 4.92	13.35 ± 2.75	72.43 ± 13.60	42.30 ± 8.05
t	—	0.026	4.447	0.009	7.296	0.032	5.672	0.057	5.709
P	—	0.979	<0.001	0.993	<0.001	0.975	<0.001	0.098	<0.001

## Data Availability

The simulation experiment data used to support the findings of this study are available from the corresponding author upon request.
